The article "An Empirical Analysis of Mental Health and Social Support in the Elderly of Different Age Groups: A Survey and Analysis of Data from China" was retracted in 2024. Reasons: signs of a paper mill; suspected computer-generated content; unreliable results or conclusions; lack of ethics approval or compliance.

# An Empirical Analysis of Mental Health and Social Support in the Elderly of Different Age Groups: A Survey and Analysis of Data from China

**DOI:** 10.1155/2022/8152971

**Published:** 2022-06-06

**Authors:** Huiyuan Qiang, Lin Liu

**Affiliations:** College of Marxism, Nanjing University of Aeronautics and Astronautics, Jiangsu, Nanjing 210016, China

## Abstract

To explore the effects of social support on the mental health of older adults in different age groups in China, and to provide reference for the development of social support policies to promote the mental health of older adults in China. This paper uses a random sampling method to conduct a questionnaire survey of 3,000 older adults aged 60 years or older in Nanjing and a dichotomous logistic regression model for empirical analysis. The two dimensions of mental health and social adjustment were used to measure the mental health status of the elderly. The results showed that the overall mental health status of the elderly in Nanjing city was more optimistic, and the nonempty nesters with male gender, higher education level, and partners were generally healthier; objective and subjective support had significant positive effects on the mental health of middle and high aged elderly, while the utilization of support had more significant effects on the health of low-aged elderly. This paper proposes that government departments should develop a localized elderly support system and social support policies adapted to the actual situation in Nanjing according to the quantitative distribution and demand characteristics of the mental health of elderly people in different age groups. The study is structured as follows: the second part contains data sources and statistical methods. The third part is the analysis of empirical results. The fourth part is the discussion and conclusion part of the article.

## 1. Introduction

In recent years, with the continuous promotion of Health China strategy, improving the health of the population has become an important research topic in the field of public health. At the same time, with the increasing trend of aging in China, the health of the elderly has become the focus of attention of all sectors of society in China. According to the forecast data of “China's Population Aging Development Trends and Policies” released in 2020, by 2022, the proportion of China's elderly population aged 65 and above will reach 14%, which will far exceed the World Health Organization's judgment standard for aging (7%) [1]. This data shows that aging will be a difficult problem for China to face and overcome in the future. In this context, how to improve the health of people in the coming years through various means has become the focus of academic attention. Current research studies the health status of older adults in terms of physical and mental health and examines the effects of residential environment, financial resources [2], health insurance [3], physical activity [4], health awareness [5], and community groups on the health of older adults [6]. However, social support, as an important social instrument in addition to government support, has a very important impact on promoting the physical and mental health of the population. Based on this, this paper explores the influence of social support on the mental health of elderly people in different age groups in Nanjing from the perspective of social support, with a view to providing reference for local departments to formulate health care policies and improve the mental health of elderly people.

## 2. Data and Methods

### 2.1. Data Source

From March 2021 to September 2021, we randomly selected 3,000 people aged 60 and above in Nanjing area (Xuanwu District, Qinhuai District, Gulou District, Pukou District), and the recovery rate reached 92.4%, 2522 valid questionnaires were recovered, and the effective rate was 91%. Inclusion criteria: (i) basic recognition ability; (ii) positive and serious attitude towards the questionnaire. The elderly was classified into three age groups: low (60-69 years old), middle (70-79 years old), and high (80 years old and above). Among the valid questionnaires, there were 1,027 low-aged seniors, 892 middle-aged seniors, and 603 low-aged seniors; 1,322 men and 1,200 women; 192 seniors did not go to school, 953 in elementary school, 882 in junior high school, 382 in high school or junior college, and 113 in college and above; 1,896 had partners and 626 did not; 1,398 were empty nesters and 1,124 were nonempty nesters.

### 2.2. Methods

The study was conducted by using a customized basic information scale, a social support scale, and a modified elderly health scale for different age groups in Nanjing city. The relevant questionnaires were designed according to the scale: one was customized with basic information about the elderly: gender, age, marital status, and education level. The second is the social support scale: this scale consists of 10 entries in three dimensions: objective support (3 entries), subjective support (4 entries), and the degree of utilization of social support (3 entries) [7]. A score [2–5, 8] was assigned to each dimension. The score for social support was a total of three dimensions [3–7, 9–16], with higher scores indicating higher levels of social support. The third is the improved health scale for older adults: the scale has 73 entries in 12 factors, including physical health, mental health, and social adjustment dimensions, including 29 entries in 5 factors for physical health, 18 entries in 3 factors for mental health, and 26 entries in 4 factors for social adjustment. Each dimension is scored [2–5, 8], with higher scores indicating better health for older adults.

### 2.3. Statistical Analysis

Based on the valid data obtained from the questionnaire, statistical analysis was performed in an Excel sheet, and the data were analyzed descriptively using SPSS 22.0 software for frequency and mean ± standard deviation. We also performed a stepwise multiple linear regression analysis of the relationship between social support and elderly health using Stata 15.0 software [9].

## 3. Results

### 3.1. Social Support Scores of Older Adults in Different Age Groups

The study found that the total social support score for the elderly in Nanjing was 9.01 ± 0.94. As shown in Table 1 for the three dimensions of social support, objective support scores were low, and subjective support and utilization of support scores were high. Subjective support tended to increase more significantly with age, and senior citizens scored better than other age groups in terms of their use of support. The scores of each age group are shown in Table 1.

### 3.2. Comparison of Health Scores of Older Adults in Different Age Groups

As shown in Table 2, the overall health score of older adults decreases significantly with age. The overall health score was 10.03 ± 0.62, which is higher than the median score of 9, indicating that the overall health of the elderly in Nanjing is more optimistic. As older adults age, their mental health improves, while their social adjustment scores gradually decrease. The detailed scores for each age group are shown in Table 2.

### 3.3. Effects of Social Support on the Dimensions of Health of Older Adults

In this paper, a stepwise regression approach is used, with the underlying information as the independent variable in the first step and the dimensions of social support included in the regression model in the second step. It can be found that △*R*^2^ increases by 7.5%, 4.8%, 6.8%, and 11.9% at this time, respectively. Models 1 through 4 used the three dimensions of health status of older adults and overall health as dependent variables, respectively. From the empirical results, it is clear that men, younger, better educated, nonempty nesters, and those with partners are generally healthier in Nanjing. In addition, objective support, subjective support, and the degree of utilization of support had significant positive effects on the health of older adults in Nanjing City, and the regression coefficients showed that objective support was most significant for the overall health of older adults. The enhancement of subjective support on the social adjustment of older adults was significantly positive at the 1% level, and the enhancement of the utilization of support had a greater impact on the mental health of older adults. The empirical results are shown in Table 3.

### 3.4. Effects of Social Support on the Health of Older Adults in Different Age Groups

Models 5 to 7 are the regression results of the effects of social support on the young, middle-aged, and elderly, respectively, with the overall health of older adults in each of the three dimensions as the dependent variable. Through stepwise regression, the second step included three dimensions of social support as independent variables based on the first step, at which point △*R*^2^ increased by 7.4%, 6.7%, and 14.4%, respectively. As shown in Table 4, lower, middle, and higher aged older adults with higher education and a partner were healthier; male lower aged older adults and nonempty nesting middle-aged older adults were healthier. In addition, social support had a significant effect on the health of older adults of all ages. The objective support had the most significant positive effect on older adults, the subjective support had a significantly positive coefficient at the 1% level for middle-aged older adults, and the increased utilization of support had the greatest effect on the overall health of lower-aged older adults. The specific results are shown in Table 4.

## 4. Discussion

### 4.1. Factors Influencing the Mental Health Status of the Elderly in Nanjing

The study showed that the total score of social support for the elderly in Nanjing was 9.01 ± 0.94, which was slightly higher than the median score of 9. The overall health score of the elderly is 10.03 ± 0.62, which is higher than the median value, indicating that the overall health status of the elderly in Nanjing is more optimistic, but there is still room for improvement. In addition, nonempty nesters who are male by gender, highly educated, and have a partner are healthier overall [10]. The empirical results show that gender has a significant impact on physical and mental health and overall health of older adults, with men having better health than women, which is consistent with the findings of Tao and Zhang's study [11]. This positive effect was more pronounced in the lower age group of older adults. Comparing the regression coefficients of the health dimensions of the elderly in Nanjing, we can find that gender has the greatest influence on the mental health of the elderly compared to physical health, while there is no significant difference in social fitness.

The health of the elderly deteriorates with age, especially for the middle-aged and the elderly, the decline of physical functions leads to the restriction of mobility, which in turn affects the mental health, as well as the negative mentality that the older you get, the less useful you are, and the degree of social adaptation decreases accordingly [12]. The effect of educational attainment on all dimensions of health was significantly positive for older adults, with greater effects on mental health and social adjustment. The reason for this is that older adults with higher education levels are more health conscious, more receptive to new things, and therefore more adaptable [13]. Nonempty nesters are healthier than empty nesters, especially in terms of mental health and social adjustment. The company of children helps the elderly to maintain a happy mood, develop an optimistic attitude, and develop social adaptability [14, 15]. In addition, the mental health of older adults with partners is better than that of older adults without partners. The mutual support of partners helps older adults to get rid of loneliness and face life more optimistically, which is an important aspect of maintaining mental health for older adults [16].

### 4.2. Social Support Is Conducive to Promoting the Mental Health of Older Adults

The social support studied in this paper is divided into three aspects: objective support, subjective support, and social support utilization. The results suggest that objective support will have a positive impact on physical health, mental health, social adjustment, and overall health of older adults. Objective support mainly refers to objective practical or visible support, and financial support is an important part of objective support. When the more objective support an older person receives, it indicates the richer monetary and material support received, which can improve the living standard of the older person to a certain extent. Older people can enjoy material life and also participate in activities of interest to them with greater peace of mind and enjoy their spiritual life, thus promoting not only the physical and mental health of older people but also their social adaptation, thus promoting the improvement of their overall health [17]. Therefore, the government can establish and improve an objective support system for the elderly to enhance their material living standards and promote their general health. Subjective support mainly refers to subjective experience or emotional support, including respect, care, and understanding for the elderly [18].

Subjective support has a significant positive effect on psychological well-being, social adjustment, and general health of older adults. It may be because with age, older adults are more experienced and more capable of psychological adjustment, which is conducive to the construction of mental health. The government can give more psychological care to the elderly, such as providing free public transportation services for the elderly and encouraging them to communicate more with their friends and relatives to enhance their mental health as well as social adaptation. Utilization of support had a significant effect on all dimensions of health as well as overall health of older adults in Nanjing, with a greater degree of effect on psychological health, social adjustment, and overall health. The higher the utilization of support, the greater the individual's proactive awareness of seeking and using outside help [19]. Older adults who choose to actively talk about their troubles are able to relieve their psychological stress in a timely manner, solve the problems they encounter, participate in activities organized by social groups, and therefore maintain good contact with the outside world, which is conducive to the development of a positive mindset and the improvement of their mental health and social fitness [20]. Therefore, the government as well as the elderly institutions can promote the general health of the elderly in Nanjing by organizing more group activities for the elderly and providing them with activity places.

### 4.3. Heterogeneity Analysis of the Relationship between Social Support and Mental Health of the Elderly

The results showed that all dimensions of social support had a significant effect on the overall health of older adults. The positive effect of objective support is more pronounced for middle-aged and older adults. This is because as older adults age, their physical functions decline, their mobility becomes weaker, they no longer have financial resources or sufficient savings of their own, and they need more outside material support in their daily lives as well as in their health care [8]. Therefore, the government can develop differentiated and objective support policies according to the actual situation of different age groups of the elderly and make full use of subsidized resources to promote the improvement of the overall health of the elderly in Nanjing. The results showed no significant effect of subjective support on the health of the younger older adults and a significant contribution to the improvement of the health of the middle and older adults. As the elderly age, they are more and more likely to feel lonely, have limited mobility, and have increased morbidity rates. Therefore, the older people need more subjective support, and the government should pay attention to the mental health of older people while strengthening objective support.

Regarding the utilization of support, it had a more significant positive effect on lower aged older adults followed by middle-aged older adults and no significant effect on higher aged older adults. The reason for this is that younger seniors are more mobile, in good physical condition, and have the ability to initiate contact and communication with the outside world, which gives them more opportunities to get help from the outside world. And as we age, our physical condition declines leading to less communication with the outside world, less frequency and initiative to seek outside help, and less need for the use of support [21]. Therefore, the government should develop an elderly support system adapted to the actual situation in Nanjing City based on the quantitative distribution and demand characteristics of elderly health in different age groups, in order to make full use of subsidized resources to maximize the overall health promotion of the elderly [22].

## 5. Conclusion

This paper empirically analyzes the effects of social support on the mental health of older adults of different ages in Nanjing, with the aim of providing a reference for the development of social support policies to promote the health of older adults. The results of the study showed that the overall mental health of the elderly in Nanjing is more optimistic, and the nonempty nesters who are male in gender have higher education level and have a partner are generally healthier. Objective and subjective supports had a significant positive effect on the mental health of middle- and high-aged older adults, while the utilization of support had a more significant effect on the health of lower-aged older adults. Government departments should develop social support policies for the elderly support system adapted to the local situation in Nanjing City according to the distribution of the number of healthy elderly people in different age groups and the characteristics of their needs.

## Figures and Tables

**Table 1:** Social support scores of older people in different age groups in Nanjing.

	Total $\bar{x}\pm s$	Low-age seniors $\bar{x}\pm s$	Middle-aged seniors $\bar{x}\pm s$	Seniors $\bar{x}\pm s$
Objective support score	2.39 ± 0.65	2.41 ± 0.65	2.42 ± 0.67	2.36 ± 0.71
Subjective support score	3.01 ± 1.12	2.84 ± 1.13	2.98 ± 1.08	3.22 ± 1.10
Utilization score for support	3.61 ± 0.92	3.57 ± 1.36	3.54 ± 0.93	3.69 ± 0.99
Total social support score	9.01 ± 0.94	8.82 ± 1.24	8.94 ± 0.93	9.27 ± 0.84

**Table 2:** Health scores of older adults in different age groups in Nanjing.

	Total $\bar{x}\pm s$	Low-age seniors $\bar{x}\pm s$	Middle-aged seniors $\bar{x}\pm s$	Seniors $\bar{x}\pm s$
Physical health score	2.81 ± 0.86	3.14 ± 0.61	3.01 ± 0.94	2.29 ± 0.88
Mental health score	3.39 ± 0.83	3.19 ± 0.71	3.26 ± 0.92	3.71 ± 0.83
Social adjustment score	3.83 ± 0.76	4.19 ± 0.72	3.84 ± 069	3.45 ± 0.71
Overall health score	10.03 ± 0.62	10.52 ± 0.69	10.11 ± 0.65	9.45 ± 0.75

**Table 3:** Effect of social support on each dimension of health of the elderly in Nanjing.

Variables	Model 1 (physical health)		Model 2 (mental health)		Model 3 (social adaptation)		Model 4 (overall health)	
	Step 1	Step 2	Step 1	Step 2	Step 1	Step 2	Step 1	Step 2
Gender	-0.04∗∗ (0.01)	-0.05∗∗ (0.01)	-0.07∗∗ (0.03)	-0.09∗∗∗ (0.03)	0.13 (0.02)	0.09 (0.02)	-0.02 (0.01)	-0.01∗∗ (0.01)
Age	-0.12∗∗∗ (0.02)	-0.13∗∗∗ (0.02)	-0.09∗∗∗ (0.02)	-0.08∗∗∗ (0.02)	-0.09∗∗∗ (0.02)	-0.08∗∗∗ (0.02)	-0.13 (0.02)	-0.09∗∗∗ (0.02)
Education level	0.04∗ (0.01)	0.03 (0.01)	0.04∗∗ (0.01)	0.06∗ (0.01)	0.14∗∗∗ (0.02)	0.12∗∗ (0.02)	0.02∗∗ (0.01)	0.03∗∗ (0.01)
Whether empty nesters	0.02 (0.01)	0.04 (0.01)	0.06∗∗∗ (0.02)	0.07∗∗∗ (0.02)	0.03∗∗∗ (0.01)	0.01∗∗ (0.01)	0.12∗∗ (0.02)	0.10∗∗ (0.02)
Marriage status	0.01 (0.01)	0.02 (0.01)	-0.03∗∗∗ (0.01)	-0.04∗∗ (0.01)	-0.01∗ (0.02)	-0.01∗ (0.02)	0.01 (0.01)	0.04∗∗ (0.01)
Objective support		0.33∗∗∗ (0.01)		0.27∗ (0.02)		0.32∗∗∗ (0.01)		0.29∗∗∗ (0.01)
Subjective support		0.03∗ (0.02)		0.19∗∗∗ (0.01)		0.21∗∗∗ (0.02)		0.16∗∗ (0.09)
Support for utilization		0.14∗ (0.01)		0.24∗∗∗ (0.01)		0.21∗∗∗ (0.02)		0.29∗∗∗ (0.01)
Cons	2.86∗∗ (0.14)	3.31∗∗∗ (0.09)	3.72∗ (0.18)	2.93∗∗ (0.16)	3.84∗∗ (0.02)	2.46∗∗∗ (0.22)	3.16∗ (0.52)	3.22∗∗∗ (0.13)
△*R*^2^	0.118	0.193	0.031	0.079	0.031	0.099	0. 193	0. 312
*F*	43.22	33.25	11.37	20.58	31.07	41.16	28.16	30.99

∗*p* < 0.1, ∗∗*p* < 0.05, ∗∗∗*p* < 0.01.

**Table 4:** Effect of social support on the health of older adults in different age groups.

Variables	Model 5 (low-age elderly)		Model 6 (middle-aged elderly)		Model 7 (senior citizen)	
	Step 1	Step 2	Step 1	Step 2	Step 1	Step 2
Gender	-0.23∗∗ (0.09)	-0.21∗∗ (0.09)	-0.28 (0.12)	-0.19 (0.12)	-0.11 (0.18)	-0.16 (0.18)
Age	0.23 (0.11)	0.19 (0.11)	-0.51∗∗∗ (0.25)	-0.49∗∗ (0.25)	-0.12∗∗ (0.31)	0.41∗∗∗ (0.31)
Education level	0.11∗ (0.12)	0.09∗∗ (0.12)	0.23∗∗ (0.09)	0.28∗∗ (0.09)	0.71∗∗∗ (0.17)	0.48∗∗∗ (0.17)
Whether empty nesters	0.39 (0.13)	-0.49 (0.13)	0.42∗ (0.21)	0.17∗∗ (0.21)	0.38 (0.15)	-0.33 (0.15)
Marriage status	0.25∗ (0.14)	0.26∗∗ (0.14)	0.35∗∗∗ (0.11)	0.45∗∗∗ (0.11)	0.32∗∗∗ (0.21)	0.55∗∗∗ (0.21)
Objective support		0.082∗ (0.11)		0.19∗∗ (0.08)		0.31∗∗∗ (0.15)
Subjective support		-0.15 (0.05)		0.29∗∗ (0.14)		0.35∗∗∗ (0.09)
Support for utilization		0.25∗∗∗ (0.11)		0.09∗ (0.15)		0.55 (0.10)
Cons	7.89∗∗∗ (1.11)	5.28∗∗∗ (0.99)	10.93∗∗∗ (1.05)	9.37∗∗∗ (1.52)	15.29∗∗∗ (1.93)	17.23∗∗∗ (1.52)
△*R*^2^	0.125	0.199	0.092	0.159	0.183	0.327
*F*	7.87	6.91	10.52	9.40	18.83	30.55

## Data Availability

The raw data supporting the conclusions of this article will be made available by the authors, without undue reservation.
